# Design and Implementation of Internet of Things Technology in College Students' Innovation and Entrepreneurship Integration System

**DOI:** 10.1155/2022/3624413

**Published:** 2022-06-10

**Authors:** Huilong Li, Xiping Sun

**Affiliations:** ^1^School of Physical Science and Technology, Baotou Teachers' College, Baotou 014030, Inner Mongolia, China; ^2^Jinmenghui Magnetic Materials Co., Ltd., Baotou 014030, Inner Mongolia, China

## Abstract

In order to improve the operation efficiency of the innovation and entrepreneurship integration system of college students, this document proposes to formulate and implement the innovation and entrepreneurship integration system of college students based on “Internet technology.” The web front end is implemented by Django technology, the back end is developed by Apache server pycharm, the database is written in Python, and the database is MySQL. The system meets the expected objectives of implementing, monitoring, and managing innovation and entrepreneurship projects. How the system realizes the functions of repeated comparison projects, easy tracking projects, and fast search, and how managers can make progress at any time. By creating different account function permissions, the system realizes the login, declaration, management, and other functions required by the users of the innovation and entrepreneurship project management system. It is very suitable for college students to improve the project application, information review, and application process. At the same time, it is helpful to supervise and select teachers and greatly improve management efficiency. The test results show that the minimum values of 30, 80, and 150 simulated users in the system performance test are 4, 5, and 7, respectively. The maximum users of the system performance test model are 30, 80, 150, 64, 284, and 398. The system performance tests are taken under the conditions of 30, 80, and 150 user bandwidth, with the results of 113/min, 104/min, and 90/min. The system basically meets the daily work management standards and fully achieves the expected system design goals. The development and use of this system are related to the development of college students' innovation and entrepreneurship project management and have a clear reference for the development of innovation and entrepreneurship project management systems similar to manage workflow in the future.

## 1. Introduction

The main challenges faced by innovation and entrepreneurship at this stage are students' innovation ability, interest in entrepreneurship training, innovation ability, motivation of professional teachers' entrepreneurship education, innovation ability, the resistance of entrepreneurship implementation mechanism, and innovation ability. Entrepreneurial projects and school activities lack innovation and entrepreneurship [1]. Therefore, how to further improve the implementation system of college students' innovation and entrepreneurship courses is a key problem faced by college students' innovation and entrepreneurship teachers [2]. Establish a coordinated, orderly, and well-structured implementation system of innovation and entrepreneurship courses for college and unversity students at at different levels of the national and provincial. Relying on the provincial college students' innovation and entrepreneurship courses, school-level college students' innovation and entrepreneurship training programs, and school-level college students' innovation and entrepreneurship training programs, leads the national college students' innovation and entrepreneurship courses “Increased innovation and entrepreneurship courses.” In recent years, the research on building an innovation and entrepreneurship platform for college students has become a hot research topic for college students. It focuses on the Internet and the features that add value to it. Several papers summarize the challenges faced by innovation and entrepreneurship in the Internet era and provide effective strategies for helping college students improve their innovation and entrepreneurship skills in the Internet era.  Figure 1 shows the overall framework of the current college student innovation and entrepreneurship project management system [3].

## 2. Literature Review

Aiming at this research problem, Cao et al. have developed a relatively perfect system by adopting a complete set of information architectures and infrastructures [4]. Yuan establish and manage the underlying hardware resource pool and provide the service resources required by the upper application through the open stack platform. It is free software and open source code project to build infrastructure as a service [5]. Yong studied the statistics of entrepreneurship data and the electronization of project materials and preliminarily completed the transformation from traditional paper projects to electronic project applications. [6]. Gao et al. entrepreneurship project management system mainly refers to the editing and publishing of innovation projects through computers, and the approval of various innovation projects through computers [7]. Damayanti et al. believe that inthe third generation of college students' innovation and entrepreneurship project management system, in the era of knowledge economy in the 21st century, how to master and maximize the use of knowledge has become the key content of innovation project management. This generation of system has powerful data processing functions, can fully integrate the files in the file system and the data in the data warehouse, and provides rich innovative project mining functions and knowledge sharing methods, gradually integrating the principles and practices of knowledge management into the daily work of each innovative project management [8]. Licite et al. believe that after more than 30 years of development, with the increasing popularity of the Internet and web technology. They pay more and more attention to the actual needs of the school and the automation of business processes, which effectively solves the island phenomenon of various information platforms within the school [9]. Liu et al. believe that the new generation can effectively cooperate with the school's information management and help the school better carry out intensive management [10]. Ianenko et al. believe that while strengthening data refinement management through application systems, there are data islands between application systems that can not realize data connection, affecting business efficiency [11]. Yan et al. refined and classified some important data, set corresponding permissions according to the use scope of different teachers and students, and different business data by standardizing the Internet behavior of end-users, by using identity authentication and other methods [12]. Barau believes that the future trend of cloud computing also increases the difficulty of network data attack methods and risk identification. Only by constantly improving the school network construction, repairing the defects of the equipment itself, and strengthening the information evaluation, can we reduce the data security risk of the information system [13]. Based on the current research, this paper introduces some key technologies used in the system, such as B/S architecture, pycharm integrated development environment, Django (Python Web Framework) technology, MySQL database, and Internet of Things authentication algorithm, which compares and analyzes these technologies, finds out the relevant technologies suitable for the system, and makes full preparations for the development of the system. Demand analysis is an important step of platform construction. Through the specific analysis of business scenarios, the business requirements of the platform can be obtained. System requirement analysis is also called software requirement analysis. The web front end is implemented by Django technology, the back end is developed by Apache server pycharm, the database is written in Python, and the database is MySQL. The development and use of this system are related to the development of college students' innovation and entrepreneurship project management and have a clear reference for the development of innovation and entrepreneurship project management systems similar to management workflow in the future.

## 3. Method

### 3.1. Relevant Technical Support

#### 3.1.1. B/S Architecture

B/S architecture, namely browser and server architecture mode, is a mode proposed after the widespread use of the web global wide area network. This mode can directly use the browser to connect and transmit data with the server. At first, many web games of this mode, which is more convenient than C/S structure. Users no longer need to download the client, and user data is also stored in the browser and server [14]. Browser is widely used in the operating system. Users can greatly improve the speed by docking data between browser and server, but there are also some problems, such as the consumption of memory will increase with time, and the optimization problem is difficult to be well solved. B/S structure is composed of three-layer structure, and it is shown in Figure 2.

The first layer is the presentation layer, which mainly shows the interactive information between users and servers at the user level. The second layer is the business logic layer, which mainly applies the business logic functions to the software functions used by users. The third layer is the data access layer, which takes data from the database after responding to the user's request [15].

The obvious disadvantages of B/S architecture are that it is weak on cross-browser. The function is weakened, there are functions that cannot be realized, and the performance is relatively low. The comparison between B/S architecture and C/S architecture is shown in Table 1.

#### 3.1.2. Pycharm Integrated Development Environment

Pycharm is a development environment that integrates multiple functions. Therefore, it can improve the efficiency of Python development [16]. It includes a complete set of Python language development tools such as code debugging, jump, project management, intelligent operation, and automatic completion of instructions [17]. Moreover, it also provides some advanced functions, such as using Django for web development.

#### 3.1.3. Django (Python Web Framework) Technology

Django adopts MTV architecture mode (i.e., model M, view v, and template T), which is an open source code of web application architecture written in Python [18]. It is a better web framework in Python, integrates many modules, and makes the connection between modules more stable.

Django has the following characteristics:

  Perfect documents: after long-term development, improvement, and consolidation, it can provide users with relatively perfect online documents, and this sort of online documents can be provided to developers to find solutions at any time, so it can improve development efficiency.
  Integrated ORM component: the model layer of Django has its own database ORM component, which is used to operate different classes.
  Type database provides a unified way [19].
  URL mapping technology: Django's mapping uses URL regular management expressions because the URL character encoding is composed of strings, which has great convenience and flexibility for developers.
  Background management system: this management system is simple and easy to operate. Users can realize background operation and web management control through a few lines of simple code and instructions [20].
  Error message prompt: if there are errors or exceptions in the process of development, debugging, and use, Django can prepare to locate the places with errors and problems and display the error information, so as to facilitate developers to modify and improve accurately and efficiently.

#### 3.1.4. MySQL Database

MySQL database is a relational database. Its highlight is open source and many people use it. It is a small and medium-sized database, but it is enough for this topic. This topic does not need a particularly large database. Alibaba Taobao used this database before 2012, so this database is sufficient for this topic. Its disadvantage is that there is no way to store and process some super large data, which does not exist in this subject [21]. MySQL database provides interfaces (APIs) for many high-level programming languages and Python used in this topic. It supports multithreaded data processing and multiCPU. Although the database is open source, it has very good security and reliability and provides a variety of data types, including common data types [22]. It has a good memory management mechanism, which can effectively prevent memory leakage and will prompt in time when memory overflow occurs. It supports all database query statements and can be used on all platforms.

#### 3.1.5. Internet of Things Authentication Algorithm

For some nodes of wireless sensor networks, the algorithm complexity of SHA-256 and other algorithms is still high, which is not suitable for terminal nodes with low processing capacity. At the same time, the old algorithms still have good performance in security. Therefore, the method adopted in this paper is still based on SHA-1 with relatively fast speed, which is also the prerequisite of sinusoidal projection authentication scheme [23]. The random number (160 bits, i.e., composed of 40 hexadecimal numbers) is issued to the node by the platform. After the node receives it, the independent variable value of sinusoidal projection is calculated with the node key, which is the identity authentication element. The specific calculation method is as follows:

Random number (expressed as 40 hexadecimal numbers):

(1) $$\begin{array}{c} R=k_{1}k_{2}k_{3}\text{…}k_{40},\\ SR=\text{SHAI}\left(R\right),\\ \text{SHAI}\left(R\right)=K_{1}K_{2}K_{3}\text{…}K_{40}. \end{array}$$

Each *k*_*n*_ and *K*_*n*_ represent a hexadecimal number.

Keys:

(2) $$\begin{array}{c} \text{key}=s_{1}s_{2}s_{3}\text{…}s_{40},\\ {\text{key}}^{\prime }\left(a\right)=s_{a}s_{a+1}\text{…}s_{40}s_{1}s_{2}\text{…}s_{a-1},\\ {\text{key}}^{\prime }\left(b\right)=s_{b}s_{b+1}\text{…}s_{40}s_{1}s_{2}\text{…}s_{b-1}. \end{array}$$

The key transformation value after hash transformation is as follows:

(3) $$\begin{array}{c} {\text{skey}}^{\prime }\left(a\right)=\text{SHAI}\left({\text{key}}^{\prime }\left(a\right)\right),\\ \text{SHAI}\left({\text{key}}^{\prime }\left(a\right)\right)=S_{a}S_{a+1}\text{…}S_{40}S_{1}S_{2}\text{…}S_{a-1},\\ {\text{skey}}^{\prime }\left(b\right)=\text{SHAI}\left({\text{key}}^{\prime }\left(b\right)\right).\\ SHAI\left({\text{key}}^{\prime }\left(b\right)\right)=S_{b}S_{b+1}...S_{40}S_{1}S_{2}...S_{b-1}. \end{array}$$

Among them, *s*_*n*_ and *S*_*n*_ also represent a hexadecimal number. A and B are the displacement identification of the key, which circularly displaces the key by *a* bits and *b* bits.

(4) $$\begin{array}{c} \text{a,b}\in \left[\text{0, }40\right). \end{array}$$

Then, in the sine projection independent variable,

(5) $$\begin{array}{c} x_{0}=SR=K_{1}K_{2}K_{3}\text{…}K_{40},\\ x_{1}=\text{SHAI}\left(R\right)⊕\text{SHAI}\left({\text{key}}^{\prime }\left(a\right)\right),\\ \text{SHAI}\left(R\right)⊕\text{SHAI}\left({\text{key}}^{\prime }\left(a\right)\right)=SR⊕{\text{skey}}^{\prime }\left(a\right),\\ SR⊕{\text{skey}}^{\prime }\left(a\right)=\left(K_{1}⊕S_{a}\right)\left(K_{2}⊕S_{a+1}\right)\text{…}\left(K_{40}⊕S_{a-1}\right),\\ \left(K_{1}⊕S_{a}\right)\left(K_{2}⊕S_{a+1}\right)...\left(K_{40}⊕S_{a-1}\right)=\alpha_{1}\alpha_{2}\text{…}\alpha_{40},\\ x_{2}=\text{SHAI}\left[R⊕{\text{key}}^{\prime }\left(b\right)\right],\\ \text{SHAI}\left[R⊕{\text{key}}^{\prime }\left(b\right)\right]=\text{SHAI}\left[\left(k_{1}⊕s_{b}\right)\left(k_{2}⊕s_{b+1}\right)\text{…}\left(k_{40}⊕s_{b-1}\right)\right],\\ \text{SHAI}\left[\left(k_{1}⊕s_{b}\right)\left(k_{2}⊕s_{b+1}\right)...\left(k_{40}⊕s_{b-1}\right)\right]=\beta_{1}\beta_{2}\text{…}\beta_{40}, \end{array}$$

where ⊕ means that the number of digits on both sides of the equal sign is consistent and any carry generated is omitted. The complete independent variable (composed of 40 hexadecimal numbers) is shown in the following equation:

(6) $$\begin{array}{c} X=X_{1}X_{2}\text{…}X_{40}. \end{array}$$

### 3.2. System Functional Requirements

The functional requirements analysis of the system is to clarify the needs of target customers and build the implementation architecture after in-depth understanding and analysis. Combined with relevant technical methods, establish an abstract model for the target, refine the realization of various functions, establish a logical model, design the system according to the architecture, and complete the realization of the system [24]. The functional structure of the system is shown in Figure 3.

Generally, it can be divided into four basic modules as shown in Figure 3.

System manager is the authority and responsibility of system administrator and project administrator. It mainly assigns its own permissions to other users, creates accounts for instructors and students, and adds project administrators, judges, teachers, and approvers [25]. Message notification management is mainly used to remind users of the link of the project, the items that need your approval or review, or the latest notifications. Online declaration management is the process of project declaration. Its process can be divided into project information registration, project declaration, project audit, project redeclaration, project modification, etc. Project management has two parts: one is to further improve or resubmit and modify the projects under application, the other is how to conduct an interim inspection and closing of the projects under application, and the contribution of everyone in the team [26].

## 4. Results and Analysis

### 4.1. Database Design

Meeting the needs of users is the basic requirement of system database design. According to the actual operation environment of the system, build an efficient storage database mode. The core of system architecture and design is the design of database, and relevant programs, which are created through database application system. At the same time, data maintenance must follow the one-to-one design principle. In order to avoid repeated naming, we must abide by the unique naming principle and the two-way use principle to obtain data information.

#### 4.1.1. Entity Diagram

We can clearly get the interaction relationship between them and display it through the entity contact diagram (E-R diagram), so as to determine the corresponding relationship between their entities.

According to the information entity, there can be user basic information entity, project basic information entity, project member basic information entity, project application form information entity, interim inspection information entity, acceptance information entity, and project review information entity. Therefore, they should be distinguished when making database tables, and their entity attributes are also different. Entity information is shown in Figures 4–6.

#### 4.1.2. Database Table Structure Design

The design of database table structure can reflect the logical relationship among entity attributes. The quality of the design directly affects the experience of using the system. The basic structure of the system is shown in Tables 2–5.

### 4.2. System Test

#### 4.2.1. Overall System Test

The overall test of the system is the test method with the largest granularity among all tests. It is the last step of the online system. It is mainly to check whether the output results meet the expected objectives. This test method is more intuitive, so it is tested manually, as shown in Table 6.

#### 4.2.2. Test of Some Functional Modules

Understand the characteristics and operation mode of the system, determine the key points of the functional module test, and then test each functional module of the system one by one to see whether the test results meet the expected objectives, and then determine the system error problem. The following is the test method of user login function module, which is tested by the PyUnit test framework. Other function modules can be tested according to the test method of login module.  Table 7 takes the login function module as an example to analyze the function test. Through the test of some special characters, MySQL security test, and illegal verification test, the security of system operation can be determined only after the test of all function modules.

#### 4.2.3. Safety Test

The system security test is about whether the system can intercept illegal access and malicious attacks. The system is configured with many functional permissions, and the functions that each permission can make are also different. All permissions are also encrypted by the MD5 encryption algorithm, as shown in Table 8.

#### 4.2.4. Compatibility Test

For multiple versions of different browsers, such as IE7.0 to IE10, the stable operation state of each interface of the system and the normal use of functional modules are shown in Table 9.

#### 4.2.5. Performance Test

The innovation and entrepreneurship training project management system simulates 3080150 users, respectively, by using the Load Runner test tool. By running the system, users can read data, check the response time of each functional module, record the appropriate time, judge whether the system performance meets the expected requirements, and calculate the system response speed. The system performance test results are shown in Figures 7–9. As shown in Figures 7–9, the performance of the system is relatively stable.

Through the test of the whole system and each functional module, it can be seen from the test result form that the system basically meets the standard of daily work management and fully meets the expected goal of system design.

## 5. Conclusion

This paper introduces the design and implementation of the Internet of Things technology in the college students' innovation and entrepreneurship integrated system and introduces some key technologies used in the B/S architecture, pycharm integrated development environment, Django (Python Web Framework), and other systems. MySQL database, Internet of Things verification algorithm, compare and analyze these technologies, find relevant technologies for the system, and provide sufficient preparation for system development. This paper discusses the business requirements, system construction principles, construction scope, purpose, and construction scheme of the college students' innovation and entrepreneurship project management system. Demand analysis is an important step in building a platform. Through special analysis of business options, the business requirements of the platform can be obtained. System requirements analysis is also known as software requirements analysis. Database development: through the inspection of the entire system and each functional module, it can be seen from the test result table that the system basically meets the daily work management standards and fully meets the expected system design goals. Later improvement combined with school innovation and entrepreneurship, on the one hand, students can understand the impact of previous business projects, which is of great benefit to students participating in the project. On the other hand, if teachers think that the projects proposed by students are practical, they can propose to implement the projects on the basis of innovation and entrepreneurship of college students.

## Figures and Tables

**Figure 1:** Overall framework of college students' innovation and entrepreneurship project management system.

**Figure 2:** Three-tier architecture of B/S.

**Figure 3:** System function structure.

**Figure 4:** User entity diagram.

**Figure 5:** Entity diagram of project information.

**Figure 6:** Entity diagram of project member information.

**Figure 7:** System performance test simulated user minimum value.

**Figure 8:** Maximum value of simulated users in the system performance test.

**Figure 9:** System performance test simulated user throughput.

**Table 1:** Comparison between B/S and C/S.

Framework	C/S	B/S
Establish foundation	LAN	Wide area network
Install	Installation required	Just a browser
Pressure	High client pressure	High server pressure
Others	The cost of upgrading and maintenance is high, which is not affected by the network speed. It is safer and cannot share resources with other computers when the network is disconnected.	It is more adaptable, affected by the network speed, not safe enough, pays more attention to access speed, has strong sharing, convenient business expansion, simple maintenance, and large compatibility problems.

**Table 2:** User table.

Field name	Type	Remarks
User name	Int[50]	User name
E-mail	Varchar[50]	E-mail
Phone	Int[50]	Phone
Role	Varchar[50]	Role
Level	Int[50]	Level
Name	Varchar[50]	Name
Identity	Int[50]	Identity
Company	Varchar[50]	Company
Introduction	LONGTEXT	Introduction

**Table 3:** Innovation projects.

Field name	Type	Foreign key	Remarks
Title	Varchar[50]		Title, primary key
Pro_id	Int[50]	Yes	Item no.
Ori	Varchar[50]		Source
BG	LONGTEXT		Project background
Con	LONGTEXT		Project introduction
Inn	LONGTEXT		Innovation or originality
Plane	LONGTEXT		Prospectus
Fund	LONGTEXT		Funds
Pre	LONGTEXT		Expected results
Comment	LONGTEXT		Instructor comments
Opinion	LONGTEXT		Review comments
Mat	LONGTEXT		Project maturity

**Table 4:** Entrepreneurial projects.

Field name	Type	Foreign key	Remarks
Title	Varchar[50]		Title, primary key
Pro_id	Int[50]	Yes	Item no.
Ori	Varchar[50]		Source
Entry	Varchar[50]		Enterprise mentor
BG	LONGTEXT		Project background
Con	LONGTEXT		Project introduction
Inn	LONGTEXT		Innovation or originality
Product	LONGTEXT		Product
Plane	LONGTEXT		Prospectus
Fund	LONGTEXT		Funds
Pre	LONGTEXT		Expected results

**Table 5:** Project management table.

Field name	Type	Remarks
Pro_id	Int[50]	Item number, primary key
Parti	LONGTEXT	Participants
PIvo	Varchar[50]	Closing certificate no.
Award	Varchar[50]	Award level
Achieve	LONGTEXT	Achievements
Mid	LONGTEXT	Interim assessment report
Conclusion	LONGTEXT	Closing material
Delay	LONGTEXT	Extension application
Change	LONGTEXT	Project change
Other	LONGTEXT	Other instructions

**Table 6:** Overall system function test.

Function name	Test description	Whether the test passes
Permission assignment function	After allocation, the user obtains this permission.	Yes
Add user functions	After adding, the user can log in to the system.	Yes
Delete user function	After deletion, the user cannot log in to the system.	Yes
Modify information function	The user's permission and password can be modified.	Yes
Project declaration function	After completing the declaration, it will be sent to the next step for review.	Yes
Mid-term inspection or closing upload function	Various materials for mid-term inspection can be uploaded.	Yes
Approval function	After approval, it can reach the next link or return to the applicant.	Yes
Review function	The review results can be displayed to the applicant.	Yes
View history item function	Users can view or search.	Yes
Export function	Users can export the required materials.	Yes

**Table 7:** Partial test of the login function module.

Serial number	Use case level	Input	Operation steps	Expected results
1	Important	Do not enter mailbox and password	Click the login button	The system prompts “mailbox or password cannot be empty.”
2	Commonly	No e-mail, only password	(1) Mailbox is empty (2) Password is not empty	Prompt “incorrect mailbox format”
3	Commonly	The mailbox is not empty, but no password has been entered.	(1) Correct e-mail format (2) No password entered (3) Click login	Prompt “password cannot be empty”
4	Commonly	Enter the correct e-mail address and password.	(1) Enter the correct mailbox (2) Enter the correct password (3) Finally, click the login button	Prompt “login succeeded”
5	Commonly	Enter e-mail correctly and password incorrectly.	(1) E-mail input (2) Input the wrong password (3) Click login	Prompt “login failed”
6	Commonly	Cursor in and out experience (with and without content)	(1) Enter e-mail (2) Enter password (3) Click login	Prompt “login failed”

**Table 8:** Safety test.

Test content	Basic requirements	Test situation	Test passed Pass or not
Application level security	Including access to data or business functions. Under the expected security, operators can only access specific functions and limited data of the application. During the test, determine the user types with different permissions, create each user type and verify its permissions with the transactions unique to each user type, and finally modify the user type and rerun the test for the same user.	Implementation requirements	Yes

System level security	It can ensure that only users with system access can access the application, and can only access through the corresponding gateway, including login or remote access to the system. The test is to verify that only operators with system and application access can access the system and application.	Implementation requirements	Yes

**Table 9:** Compatibility test.

Test content	Basic requirements	Test situation	Test passed Pass or not
Browser compatibility	For the current mainstream browser (including version), on the premise of ensuring that the compatibility test of the mainstream browser passes, test the nonmainstream browser (including version) to ensure the integrity of the compatibility test of the browser of the project as far as possible.	The system shows little difference in different browsers.	Yes

## Data Availability

The labeled dataset used to support the findings of this study is available from the corresponding author upon request.
